The article "MIM-Deficient Mice Exhibit Anatomical Changes in Dendritic Spines, Cortex Volume and Brain Ventricles, and Functional Changes in Motor Coordination and Learning" was published in 2019. Journal: Front Mol Neurosci.

# MIM-Deficient Mice Exhibit Anatomical Changes in Dendritic Spines, Cortex Volume and Brain Ventricles, and Functional Changes in Motor Coordination and Learning

**DOI:** 10.3389/fnmol.2019.00276

**Published:** 2019-11-15

**Authors:** Rimante Minkeviciene, Iryna Hlushchenko, Anaïs Virenque, Lauri Lahti, Pushpa Khanal, Tuomas Rauramaa, Arto Koistinen, Ville Leinonen, Francesco M. Noe, Pirta Hotulainen

**Affiliations:** ^1^Minerva Foundation Institute for Medical Research, Helsinki, Finland; ^2^A. I. Virtanen Institute for Molecular Sciences, University of Eastern Finland, Kuopio, Finland; ^3^HiLIFE - Neuroscience Center, University of Helsinki, Helsinki, Finland; ^4^Department of Computer Science, Aalto University School of Science, Espoo, Finland; ^5^Department of Clinical Pathology, Kuopio University Hospital, University of Eastern Finland, Kuopio, Finland; ^6^SIB Labs Infrastructure Unit, University of Eastern Finland, Kuopio, Finland; ^7^Neurosurgery of NeuroCenter, Kuopio University Hospital, University of Eastern Finland (UEF), Kuopio, Finland; ^8^Research Unit of Clinical Neuroscience, University of Oulu, Oulu, Finland; ^9^Department of Neurosurgery, MRC Oulu, Oulu University Hospital, Oulu, Finland

**Keywords:** dendritic spines, brain ventricles, learning, motor coordination, anxiety

## Abstract

In this study, we performed a comprehensive behavioral and anatomical analysis of the Missing in Metastasis (Mtss1/MIM) knockout (KO) mouse brain. We also analyzed the expression of MIM in different brain regions at different ages. MIM is an I-BAR containing membrane curving protein, shown to be involved in dendritic spine initiation and dendritic branching in Purkinje cells in the cerebellum. Behavioral analysis of MIM KO mice revealed defects in both learning and reverse-learning, alterations in anxiety levels and reduced dominant behavior, and confirmed the previously described deficiency in motor coordination and pre-pulse inhibition. Anatomically, we observed enlarged brain ventricles and decreased cortical volume. Although MIM expression was relatively low in hippocampus after early development, hippocampal pyramidal neurons exhibited reduced density of thin and stubby dendritic spines. Learning deficiencies can be connected to all detected anatomical changes. Both behavioral and anatomical findings are typical for schizophrenia mouse models.

## Introduction

Dendritic spines, along the dendrites of excitatory neurons, are functional units of the brain that play important roles in various cognitive functions. *In vivo* two-photon imaging in animal models has shown that dendritic spine density increases during learning (Xu et al., 2009; Yang et al., 2009; Yu and Zuo, 2011), with a strong positive correlation between the number of dendritic spines gained after learning and the performance in relevant memory tasks (Xu et al., 2009; Yang et al., 2009). Depletion of learning-induced new spines results in the loss of the memory formed (Hayashi-Takagi et al., 2015). Disease-specific disruptions in dendritic spine shape, size or number accompany a large number of neurological disorders, particularly those that involve deficits in information processing, suggesting that dendritic spines may serve as a common substrate (Penzes et al., 2011). Concurrently, alterations of cerebrospinal fluid (CSF) flow and increase in intracranial pressure are also correlated with cognitive problems. In older adults, for instance, typical symptoms of hydrocephalus – meaning enlarged brain ventricles, associated with increased CSF volume, and increased interstitial fluid – involve memory loss, progressive loss of cognitive functions, poor motor coordination or balance, as well as difficulty in walking (Williams and Malm, 2016). In fact, in addition to defects in dendritic spines, hydrocephalus is often comorbid in different neurological disorders, such as schizophrenia (Bakhshi and Chance, 2015).

The article "MIM-Deficient Mice Exhibit Anatomical Changes in Dendritic Spines, Cortex Volume and Brain Ventricles, and Functional Changes in Motor Coordination and Learning" was published in 2019. Journal: Front Mol Neurosci.

In our earlier study, we showed that, during brain development, a protein called Missing in Metastasis (MIM), also known as MTSS1, initiates new dendritic spines by locally curving the membrane of the dendrite (Saarikangas et al., 2015). In the cerebellum of MIM knockout (MIM KO) mice, Purkinje cells present a reduced number of spines and abnormal dendrites: these relate to cerebellum-dependent defects in motor coordination, as well as in an alteration of the electrophysiological properties of Purkinje Cells (Saarikangas et al., 2015; Sistig et al., 2017). Furthermore, *in vitro* studies have shown that alterations in the number of spines are also present in MIM KO hippocampal pyramidal neurons (Saarikangas et al., 2015).

In order to provide a more comprehensive picture of the cellular processes affected by MIM deficiency and of related behavioral outcomes, in the present study we performed a broader behavioral and histological analysis of MIM KO mice. We also analyzed MIM expression at different ages at different brain areas. Our data show that MIM is highly expressed in cerebellum throughout life but its expression in hippocampus and cortex decreases strongly after early development. Histological analyses revealed enlarged ventricles and decreased cortical volume, and a decreased density of thin dendritic protrusions. All these changes are associated with observed behavioral defects in learning and motor-coordination.

The article "MIM-Deficient Mice Exhibit Anatomical Changes in Dendritic Spines, Cortex Volume and Brain Ventricles, and Functional Changes in Motor Coordination and Learning" was published in 2019. Journal: Front Mol Neurosci.

## Materials and Methods

### Animals

In the present study we used MIM knock-out (MIM KO) transgenic mice on a C57Bl/6J background and littermates wild-type (WT) mice as controls. Animals were housed 2–3 mice per cage in a controlled environment (temperature 21 ± 1°C, humidity 50 ± 10%, light period 07:00 AM to 7:00 PM) and supplied with food and water *ad libitum*. Behavioral testing was performed in young animals (starting at P112 ± 14 days) and re-tested in the same mice at older age (starting at P294 ± 14 days). The behavioral tests were executed in this order (starting from the less stressful test): zero maze, open field, light/dark box, vertical grid, grip strength, rota-rod, stress induced hyperthermia, pre-pulse inhibition (PPI), hot plate, foot print, Barnes test, water maze, tube test and forced swim test. All behavioral tests were executed between 08:00 and 15:00 h. A minimum 2-day interval between tests and at least 30 min acclimatization time in the testing room before testing were respected. For all procedures experimenters were blind to the genotype.

### Behavioral Phenotyping

The following behavioral tests were carried out: anxiety level and locomotor activity (open field, zero maze, light/dark box, stress induced hyperthermia), motor coordination (rota-rod, vertical grid test, grip strength, foot print), nociception (hot plate), sensorimotor gating (PPI), learning and memory (Morris water maze, Barnes test), behavioral despair (forced swim test), and social behavior (tube test). Young group (P112 days of age) consisted of the following number of mice: wt 12 males + 12 females, MIM KO 10 males + 8 females. Aged group was the same cohort of mice, excluding three MIM KO mice which died before behavioral testing. Thus, in aged group (P294 days of age) there were 12 males WT, 12 females WT, 9 males MIM KO and 6 females MIM KO. All experiments were carried out in accordance with the guidelines laid down with the European Communities Council directive of 2010/63/EU and were approved by the County Administrative Board of Southern Finland (license number ESAVI/4943/04.10.07/2016).

#### Zero Maze

Unconditioned anxiety-like behavior was measured by the degree to which the rodent avoids the unenclosed areas of the maze. A zero-maze made from cycling corridor (an outer wall circumference of 50 cm and 5 cm wide) elevated above the floor (50 cm) and provided with two open areas and two closed areas. Mice were placed in the closed area of the maze facing a wall and allowed to explore freely for 5 min. Behavior was recorded using the EthoVision video tracking system (Noldus Information Technology, Wageningen, Netherlands). Automated tracking was used for the analysis of time spent and the number of entries to the open and closed areas.

The article "MIM-Deficient Mice Exhibit Anatomical Changes in Dendritic Spines, Cortex Volume and Brain Ventricles, and Functional Changes in Motor Coordination and Learning" was published in 2019. Journal: Front Mol Neurosci.

#### Open Field

The open field was assessed using activity monitor system (Med Associates, United States) to determine general activity levels, gross locomotion activity, and exploration habits. The animal was placed in the corner of the arena (30 × 30 cm) facing the wall and allowed to freely move for 30 min while being tracked by an automated tracking system with three planes of infrared detectors. Distance moved, velocity, vertical count, and times spent in pre-defined areas of the arena were recorded. For the analysis of anxiety behavior, the arena was divided into a central (18 × 18 cm) and a peripheral zone, and latency to enter the central zone, the distance traveled in the central zone and the total distance traveled were scored.

#### Light-Dark Box

Experimental arena (30 × 30 cm, Med Associates, United States) was divided using inserts non-transparent for visible light into two equal parts: a white open zone (illuminated at ∼550 lx) and a dark zone; light and dark areas were connected by an opening at floor level (5.5 × 7 cm). At the start of the test, the mouse is placed into the dark area and allowed to explore the experimental chamber freely for 10 min. The number of entries and the time spent in either zone was detected by infrared sensors and collected by an activity monitor system.

#### Vertical Grid Test

The mouse was placed on a horizontal wire grid (25 cm high and 22 cm wide, with 2 mm diameter wires spaced at 1 cm). The grid was turned immediately to the vertical position with the mouse facing the floor at the lower edge. Time to turn upward, to climb to the upper edge or to fall off from the grid was measured by stop-watch for 1 min maximum.

#### Grip Strength

A grip strength meter (Ugo Basile, Italy) was used to assess forelimb and all limbs grip strength. Mice were lifted and held by their tail so that their forepaws could grasp a wire grid. The mice were then gently pulled backward by the tail with their posture parallel to the surface of the table until they release the grid. The peak force applied by the forelimbs or all limbs of the mouse was recorded in gram-force (gf). Each mouse was tested five times for forelimbs and five times for all limbs and the average value obtained was used for statistical analysis.

#### Rota-Rod

For evaluation of coordination and motor learning the accelerating (from 4 to 40 rpm in 5 min) rota-rod (Ugo Basile, Italy) test was performed. Trials began by placing the mouse on an accelerating apparatus. Each trial lasted for a maximum of 6 min or ended whenever the mouse fell off the rod, and latency was recorded. Mice were tested for three trials a day (1-hour inter-trial interval) for two consecutive days.

The article "MIM-Deficient Mice Exhibit Anatomical Changes in Dendritic Spines, Cortex Volume and Brain Ventricles, and Functional Changes in Motor Coordination and Learning" was published in 2019. Journal: Front Mol Neurosci.

#### The Stress-Induced Hyperthermia (SIH) Test in Mice

This protocol has proven reliable in detecting the anxiolytic properties of test compounds or genotype susceptibility to stress (Adriaan Bouwknecht et al., 2007). In this test, SIH is quantified in mice using a rectal temperature measurement as the stressor. Rectal temperature is measured twice at a 10 min interval. Due to the stress experienced during the first temperature measurement, the temperature of the second measurement (T_2_) is ∼0.8° to 1.5°C higher than that of the first (T_1_). This difference in temperature (ΔT = T_2_−T_1_) is defined as the SIH response.

#### Acoustic Startle Test and Pre-pulse Inhibition

For the tests, mice were enclosed in a transparent plastic tube positioned in the startle chamber (diameter 4.5 cm, length 8 cm, Med Associates, United States) with a background white noise of 65 dB and left undisturbed for 5 min. Acoustic startle stimuli (20 ms white noise bursts) were presented in random order with 8–15 s between the subsequent trials. Altogether 36 trials with the following noise intensities were randomly applied: 68, 72, 75, 78, 82, 86, 90, 100, 110 dB. The startle response was recorded for 65 ms starting with the onset of the startle stimulus. The maximum startle amplitude recorded during the 65 ms sampling window was used as the dependent variable and averaged over 4 trials with given stimulus intensity.

Pre-pulse inhibition of acoustic startle response was examined 2 days after the acoustic startle response assessment in the same groups. The apparatus and basic experimental conditions were identical to those described above. Testing was performed in 12 blocks of 5 trials and five trial types were applied. One trial type was a 40 ms, 120 dB white noise acoustic startle stimulus (SS) presented alone. In the remaining four trial types the startle stimulus was preceded by the acoustic pre-pulse stimulus (PPS; white noise bursts of 68, 72, 76 or 80 dB). The delay between the onset of PPS and SS was 100 ms. The 1st and 12th block consisted of SS-alone trials. In remaining blocks the SS and PPS + SS trials were presented in pseudorandomized order such that each trial type was presented once within a block of five trials. The inter-trial interval ranged between 10 and 20 s. The startle response was recorded for 65 ms starting with the onset of the startle stimulus. The maximum startle amplitude recorded during the 65 ms sampling window was used as the dependent variable. The startle response was averaged over 10 trials from blocks 2–11 for each trial type. The pre-pulse inhibition for each PPS was calculated by using the following formula: 100−[(startle response on “PPS + SS trials”/startle response on “SS trials”) × 100].

The article "MIM-Deficient Mice Exhibit Anatomical Changes in Dendritic Spines, Cortex Volume and Brain Ventricles, and Functional Changes in Motor Coordination and Learning" was published in 2019. Journal: Front Mol Neurosci.

#### Hot Plate

During the experiment, the mouse was introduced into an open-ended cylindrical space with a floor consisting of a heated plate 52°C. The plate heated to a constant temperature produces behavioral components that can be measured in terms of reaction time to paw licking or paw shaking.

#### Footprint

To obtain footprints, the hind- and forefeet of the mice were coated with blue and red nontoxic paints, respectively. The animals were then allowed to walk along a 50 cm-long, 10 cm-wide runway (with 10 cm-high walls) into an enclosed box. All mice had three trials. A fresh sheet of white paper was placed on the floor of the runway for each run. The footprint patterns were scanned, and stride length was measured with “straight-line” tool in ImageJ between the center of the footprints. In average 7 steps were measured per one trial, excluding footprints made at the beginning and end of the run where the animal was initiating and finishing the movement, respectively.

#### Barnes Test

A circular table with a diameter of 100 cm was used. Twenty holes are located at the perimeter of the table at equal distances, each with a diameter of 5 cm. One hole only (the target hole) leads to an escape chamber in which the animal can hide. For analysis purpose maze is divided into 20 equal sectors, inner area 15 cm from the edge of the maze and used as a whole zone (Figure 1H). High illumination was used to encourage the animal’s motivation to search for the target hole. During the adaptation phase, one day before testing, the animals were placed in a cylinder around the target hole to familiarize with it and learn to enter the escape box voluntarily.

**FIGURE 1:** Impairment in spatial learning and memory in MIM KO mice. **(A)** Illustrative images of mouse trajectories in the water maze during the first and last learning trials. **(B,C)** Learning curves of the water maze task during six trials over three days (hid1–hid6). Reverse-learning curves during four trials over 2 days (rev1–rev4). Group means ± SEM are shown for the escape latency to the hidden platform. **(D,F)** A 60 s probe trial for search bias was conducted on Day 4. **(E,G)** A 60 s reverse probe trial for search bias was conducted on Day 6. Time spent in near vicinity of the platform location (target), opposite poolside platform location (opposite) or two other corresponding locations symmetrically right and left of the platform. The last trial of the water maze was with a visible platform (visbl). **(H)** Illustrative images of Barnes maze with 20 holes. An escape box was placed under one box (target). The remaining holes were numbered according to their distance from the target and the letters R (right from target) or L (left from the target). **(I)** A 90 s probe trial performed on Day 4. **(J)** A 90 s reverse probe trial performed on Day 6. Time spent in target zone or other corresponding zones around the maze is presented as group mean ± SEM.^∗^ denotes statistical significance: ^∗^*p* < 0.05, ^∗∗^*p* < 0.01, ^∗∗∗^*p* < 0.001.

The article "MIM-Deficient Mice Exhibit Anatomical Changes in Dendritic Spines, Cortex Volume and Brain Ventricles, and Functional Changes in Motor Coordination and Learning" was published in 2019. Journal: Front Mol Neurosci.

Before the start of the trial, the mouse was placed in the non-transparent cylinder in the center of the arena. After 5–10 s the cylinder was removed and the animal was free to explore the arena. If the animal entered the escape box, it was kept there for 10–15 s and then it was removed with the box. If a mouse didn’t find or enter the box in 180 s, it was taken there by hand (mouse were placed close to the entrance of the escape box). Learning phase consisted of 9 trials: 3 trials per day with 1 h between trial periods. On 4th and 6th day, the probe trials were performed. Tests were conducted with closed holes and no escape chamber. Animals were given a single 90 s trial to explore the environment. Re-learning phase consisted of six trials - following the probe test, the target hole and escape chamber were moved 180 degrees from the original target location.

Latency to reach the escape chamber, total distance traveled and mean speed was automatically calculated by EthoVision video tracking system (Noldus Information Technology, Wageningen, Netherlands).

#### Morris Water Maze

Morris water maze is used to measure the spatial learning and memory of the mice. The apparatus is a beige plastic pool with a diameter of 120 cm. An escape platform (∅10 cm) is hidden 1.0 cm below the water surface. Learning phase (Days 1–3): three 60 s trials are conducted twice/day with the hidden platform. The platform location is kept constant throughout the trials. Spatial memory phase (Day 4): 24 h after the completion of the learning phase, the ability to remember the location of the platform is tested during the first probe trial (60 s), when the platform is removed. Reverse learning phase (Days 4–6): the hidden platform is moved to the opposite quadrant, and the mouse is trained for 2 days to find it (reverse learning), as described before. 24 h after the completion of the reverse learning, spatial memory of the opposite platform’s location is assessed during the second probe trial, without the platform. A computer-interfaced video-tracking system (Noldus EthoVision XT 8.0, Netherlands) is used to calculate the escape latency (time to find a platform), and the time spent in each quadrant. Mice went through similar training and spatial memory assessing phases at both tested ages. Young animals started with the platform placed at the “target” position (Figure 1A). When retested at older age, the location of the platform was moved to the “left” position. As platforms were not located in the same position at the different age tests, old animals could not just remember the platform location from the previous trial at younger age. However, mice were already acquitted to the test and developed a searching strategy. This can justify the reason why mice were able to find the platform faster during the first trial at old than young age.

The article "MIM-Deficient Mice Exhibit Anatomical Changes in Dendritic Spines, Cortex Volume and Brain Ventricles, and Functional Changes in Motor Coordination and Learning" was published in 2019. Journal: Front Mol Neurosci.

#### Tube Test

Tube dominance test was used to evaluate social dominance and aggression. Two unfamiliar mice of the same sex but different genotypes were released into opposite ends of a clear, narrow tube (30 × 3.8 cm inner diameter). The animals interact in the middle of the tube, with the more dominant animal, showing a prominent aggressive behavior, that forces the opponent out of the tube. Every round ends when one of the mice is completely out from the tube: the mouse that had all four paws out of the tube was declared the loser while the animal remaining inside the tube was the winner. Matches lasting more than 2 min or in which animals crossed over each other were not scored. The number of wins is reported as a percentage of the total number of rounds (Figure 2I). Each mouse had 7–10 rounds, every round with new unfamiliar opponent.

**FIGURE 2:** MIM KO mice exhibit altered behavior in various tests. **(A–C)** MIM KO mice had reduced anxiety and spent more time exploring the open arms of zero maze **(A)**, the center of the open field arena **(B)** and the light compartment of light/dark test **(C)** compared to WT littermates. **(D–G)** MIM KO mice exhibited motor coordination impairment in vertical grid test - representative picture of mouse climbing to the top of the grid **(D)** and time taken to climb to the top of the grid **(E)**, grip strength - five trials average was compared between groups **(F)**, latency to fall on the rota-rod task **(G)**. **(H)** Pre-pulse inhibition defect in MIM KO mice. **(I)** Percentages of the wins in the tube test. ^∗^ denotes statistical significance: ^∗^*p* < 0.05, ^∗∗^*p* < 0.01, ^∗∗∗^*p* < 0.001.

#### Forced Swim Test

Mice were placed in a glass cylinder (18 cm wide × 27 cm deep) filled with 23 - 25°C water. Behavior was recorded using a Samsung SMX-F300BP camera (Suwon, South Korea) for 6 min. Time spent immobile (motionless or only little movements to prevent sinking) was scored for three 2 min-periods.

### Histology

Morphological analysis of cells in the CA1 (cornu ammonis area 1) in mice hippocampus was performed for fixed brains expressing lentivirally transduced GFP construct. The virus was injected directly in the hippocampus at age P378, after the last behavioral test (WT *n* = 5 females + 5 males; MIM KO *n* = 5 females + 5 males) and brains were collected after 2 weeks. For that, mice were anesthetized and transcardially perfused using 50 ml cold PBS, followed by 50 ml cold 4% paraformaldehyde in PBS. Brains were postfixed overnight in 4% formaldehyde in PBS at 4°C, cryoprotected using a 10 – 20 – 30% sucrose-PBS gradient over 3 days, frozen in Tissue-Tek OCT (Sakura), and stored at −80°C before cutting. 35 μm thick sections were cut using a cryostat at −20°C, and stored in antifreeze solution (Hoffman et al., 2008). For staining, transfected sections were incubated with the primary anti-GFP antibody (1:500; Roche) overnight at 4°C. Next day sections were incubated in Alexa Fluor-594-conjugated anti-rabbit secondary antibody (1:1000; Invitrogen) for 2 h and mounted on glass coverslips using Fluoromount medium (Thermo Scientific). From the same animals one series of slices (every 10th through the brain) was stained with DAPI for ventricle size analysis. In addition, for cilia density analysis, 3–5 slices per animal encompassing the 3rd ventricle or the aqueduct were stained with the primary anti-acetylated-tubulin antibody (1:500; Sigma-Aldrich), overnight at +4°C. Next day sections were incubated in Alexa Fluor-488-conjugated secondary antibody for acetylated-tubulin (1:1000; Invitrogen) for 2 h, then co-stained with DAPI and mounted on glass coverslips using Fluoromount medium (Thermo Scientific). DAPI stainings were imaged with 3DHISTECH Pannoramic 250 FLASH II digital slide scanner and cilia were imaged with confocal microscope.

The article "MIM-Deficient Mice Exhibit Anatomical Changes in Dendritic Spines, Cortex Volume and Brain Ventricles, and Functional Changes in Motor Coordination and Learning" was published in 2019. Journal: Front Mol Neurosci.

For the evaluation of MIM expression by Western blot and immunohistochemistry (Figure 3), separate groups of animals were used: post-natal day P7 (*n* = 4 WT and *n* = 2 MIM KO mice), P26 (*n* = 2 WT and *n* = 5 MIM KO mice), P117 (*n* = 4 WT and *n* = 5 MIM KO mice), P186 (*n* = 2 MIM KO mice) and P328 (*n* = 1 WT mouse) (not all results are shown).

**FIGURE 3:** MIM expression in the brain. **(A)** Western blot data show that the MIM protein is not expressed in MIM KO mouse brain, and in WT P7 mice the highest MIM expression is in the cerebellum, while hippocampi and cortices have a lower MIM expression. In SDS-PAGE gel, MIM protein runs above 100 kDa size marker, around 115 kDa, whereas actin runs by 42 kDa. All samples, 35 μg of protein. **(B)** Cortex, hippocampus and cerebellum samples of 2 P7 WT mice, 2 P26 WT mice, 3 P117 WT mice and 1 P328 WT mice were run on SDS-PAGE gel and blotted against MIM and actin. MIM is expressed through the mouse life in cerebellum whereas in hippocampus and cortex it is expressed at higher amount only at P7. Cerebellum samples 40 μg, Cortex and hippocampus samples, 80 μg of protein. **(C–J)** Sagittal WT and KO brain sections stained for MIM **(D,F,H,J)** and counterstained for DAPI **(C,E,G,I)**. Shown are brain sections of P7 **(C–F)** and P117 **(G–J)** mice. Scale bars: 1000 μm. **(K–N)** Cerebellum **(K,M)** and hippocampus **(L,N)** in higher magnification from same sections as shown in panel **C–J** at same intensity to visualize MIM expression in Purkinje cells and granule cells in cerebellum **(K,M)** and in pyramidal and granule cells in hippocampus **(L,N)** at different ages (P7, P117). Scale bars: 100 μm.

From each mouse brain, the left hemisphere was used for immunohistochemical analysis, while the right hemisphere was dissected for Western blot analysis. Animals were anesthetized and transcardially perfused using 50 ml cold PBS. Cortex, hippocampus, and cerebellum from the right hemisphere were fast frozen in liquid nitrogen and stored at −80°C for Western blot. The left-brain hemisphere was fixed with 4% PFA for 3 days, followed by 70% ethanol for 3 days (every day refreshing solutions) and then paraffinized during 10-hour, following the adult mouse brain program on Logos One, Fully Automated Innovative Tissue Processor (Milestone Medical, Italy). Then 5 μm sagittal sections were cut for following analyses. For staining, sections went through deparaffinization and rehydration, antigen retrieval (12 min boiling in a microwave in 0.01 M citrate buffer pH 6.0), and eventually stained first with anti-MIM (1:500; Novus Biologicals) and anti-MAP2 (1:500; Millipore) overnight at 4°C. Next day, sections were incubated in Alexa Fluor-647-conjugated anti-rabbit secondary antibody (secondary for MIM, 1:1000; Life Technologies) and with Alexa Fluor-568-conjugated anti-chicken antibody (secondary for MAP2, 1:1000; Invitrogen) for 2 h and mounted with glass coverslips using Fluoromount medium (Thermo Scientific). Brain slice images were generated using 3DHISTECH Pannoramic 250 FLASH II digital slide scanner.

### Confocal Imaging and Dendritic Spine Analysis

Imaging was performed on a Zeiss LSM780 inverted confocal microscope. A 63 × 1.4 NA oil immersion objective lens and Immersol 518F (Zeiss) immersion oil were used. 35 μm thick slices were imaged first with low magnification (Figure 4A) to select dendrites for dendritic spine analysis. We used relatively thin slices to improve the imaging quality of confocal microscope. Thinner slices give less background staining and less “out of focus” dendrites to images, which interferes the dendrite and spine detection of the dendrite of interest. Imaged and analyzed dendrites were apical 1st or 2nd branch dendrites, never the primary dendrite and never the very distal ends of dendrites. Imaged dendrites were selected from areas that were far away from each other so that it was a high probability that they present different neurons. For the analysis of spine density and morphology, tiff image files comprising z-stacks of 20–30 optical sections per dendritic segment were directly processed with NeuronStudio, a software package specifically designed for spine detection and analysis (Rodriguez et al., 2008). The voxel size of the images was 0.066 × 0.066 × 0.2–0.3 μm. After modeling of the dendrite surface, default parameters of the software were used to classify spines based on their morphology; protrusions with a minimum volume of 5 voxels (0.020 μm^3^), length between 0.2 and 5 μm, and a maximal width of 3 μm were retained as spines. After modeling the dendrite surface, the spines were auto-detected and classified as “mushroom,” “thin,” or “stubby” by the software. Following the default settings of the program and the empirical classification rule defined by Rodriguez et al. (2008), spines with a minimum head diameter of 0.35 μm and a minimum head vs. neck diameter ratio of 1.1 were classified as mushroom spines. Non-mushroom spines with a minimum volume of 10 voxels (0.040 μm^3^) were classified as stubby spines. All other spines were considered thin. The model was then corrected manually: the protrusions missed by the algorithm were added and classified, the false labeling of other structures as spines was removed. Similar length of dendrite was measured from each animal.

The article "MIM-Deficient Mice Exhibit Anatomical Changes in Dendritic Spines, Cortex Volume and Brain Ventricles, and Functional Changes in Motor Coordination and Learning" was published in 2019. Journal: Front Mol Neurosci.

**FIGURE 4:** Reduced number of thin and stubby spines in the hippocampus of MIM KO mice. **(A)** Representative picture of lentiviral transfection in the CA1 area of the hippocampus. **(B,C)** Dendrites of CA1 pyramidal hippocampal neurons expressing GFP for dendritic spine analysis. Scale bars: 5 μm. **(D)** Quantification of spine morphology reveals a decreased number of stubby and thin spines without altering the total spine density. Spine density of thin, mushroom, and stubby spine morphologies: WT = 0.33 thin, 1.20 mushroom, 0.17 stubby, total density 1.70 spines/μm; MIM KO = 0.27 thin, 1.31 mushroom, 0.08 stubby, total density 1.66 spines/μm. Data represent *n* = 9 (WT) animals, 39.88 ± 1.08 μm of dendrite per animal; *n* = 9 (MIM KO) animals, 32.35 ± 1.51 μm of dendrite per animal. ^∗^ denotes statistical significance: ^∗∗^*p* < 0.01.

### Cilia Length and Density Analysis

Imaging was performed on a Zeiss LSM880 inverted confocal microscope. A 63 × 1.4 NA oil immersion objective lens and Immersol 518F (Zeiss) immersion oil were used to image the fixed mouse brain slices. The slices were stained for acetylated tubulin and DAPI. To measure the cilia length, for each animal, we obtained 10–18 z-stacks of 6–21 optical sections with a 0.5 μm step in the z-axis and a pixel size of 0.044 × 0.044 μm. To measure the cilia density, for each animal, we obtained 8–18 z-stacks of 6–23 optical sections with a 0.5–1 μm step in the *z*-axis and a pixel size of 0.22 × 0.22 μm. Images were taken along the ventricle walls.

Image files were processed with Fiji software (Schindelin et al., 2012, 2015). First, 3D image data was converted to 2D using Z-projection based on the maximum intensity of the acetylated tubulin staining signal. To measure the density of cilia for each image we measured the length of the ventricle edge shown using a “segmented line” tool, and the number of cilia was determined by marking each cilium tip with a “multi-point” tool. Then the density was calculated for each image as the number of cilia divided by the length of the ventricle edge. To assess the length of cilia for each image we measured the length of 5 to 10 visible cilia with a “segmented line” tool and the median value was taken as a representative for the image.

### Western Blotting

Hippocampus, cortex, and cerebellum of WT and MIM KO mice were first homogenized and lysed using Ultra-Turrax in RIPA buffer (50 mM Tris–HCl pH = 7.4, 1% NP-40, 0.25% sodium deoxycholate, 150 mM NaCl, and 1 mM EDTA) in addition to the 1% sodium dodecyl sulfate (SDS) and protease and phosphatase inhibitor cocktail (Roche). The protein concentration was estimated by using BCA Protein Assay (Thermo Fisher Scientific). 35 μg of protein of all samples for Figure 3A, and 40 μg of protein of cerebellum samples and 80 μg of protein of cortex and hippocampus slices for Figure 3B, were run on 10% SDS-PAGE gels. Gels were then blotted on polyvinylidene difluoride (PVDF) membrane following the manufacturer’s protocol. The membrane was then blocked for 1 h in 5% milk in TBS - 0.1% Tween 20 (TBS-T) at room temperature. The membrane was incubated in primary antibody against MIM (Rabbit, 1:1000, Novus Biologicals) diluted in 5% milk in TBS-T overnight at 4°C. The following day, the membrane was washed three times with TBS-T and then incubated in secondary antibody (anti-rabbit, 1:2500, Invitrogen) for 1 h at room temperature. After washing three times with TBS-T, the membrane was developed using Enhanced Chemiluminescence (ECL) reagent (Thermo Scientific) according to the manufacturer’s protocol.

The article "MIM-Deficient Mice Exhibit Anatomical Changes in Dendritic Spines, Cortex Volume and Brain Ventricles, and Functional Changes in Motor Coordination and Learning" was published in 2019. Journal: Front Mol Neurosci.

### *In vivo* Longitudinal MRI

A separate cohort of mice was used for MRI analyses and Evans Blue (EB) injections. MRI scans were acquired in 7 WT mice (3 females and 4 males) and 7 littermate MIM KO mice (4 females and 3 males) during a 2-month-long follow up study. Scans were acquired once per month at post-natal days P112, P140, and P168. In five mice (2 females WT, 1 female MIM KO, and 2 males WT) MRI scans have been performed also at post-natal day P84. MRI data were collected at 7T (Bruker Pharmascan, Ettlingen, Germany) using 3D T2-weighted Fast Spin-Echo sequence (RARE, repetition time 1.5 s, effective echo time 48 ms, 16 echoes per excitation) and 100 μm isotropic resolution (field of view 25.6 mm × 128.8 mm × 9.6 mm). Acquisition matrix was 128 × 256 × 96. Images were acquired with the subject under isoflurane anesthesia (5% for induction, 1.0–1.5% for maintenance, in a 70/30 N_2_O/oxygen gas mixture, 1 L/min). The average acquisition time was 50 min. The pressure sensor was used to monitor the respiratory rate, and respiratory-gating was used to minimize motion artifacts.

### Ventricular Volume Measurement

Three-dimensional ventricles reconstructions were extracted by a single operator blinded to the genotype of the analyzed animals, by manually outlining regions of interest (ROIs) in each axial image, using the ROI tool in AEDES, a free in-house written Matlab program developed at University of Eastern Finland. ROIs were drawn according to the Franklin and Paxinos (2007) mouse anatomical atlas (3rd edition), including the lateral, 3rd and 4th ventricles and the aqueduct. Measured brain area was the full area of a brain slice, including the areas of all ventricles.

### Cortical Thickness Measurement

Cortical thickness measurements were conducted in four areas on T2-weighted images acquired at post-natal days P112, P140, and P168, using ImageJ (image processing and analysis in Java), as previously described: the primary somatosensory cortex barrel field (S1BF), the dorsal area of the auditory cortex (AuD), the dorsolateral entorhinal cortex (DLEnt) and the striatum have been analyzed. MRI images were segmented based on Franklin and Paxinos (2007) mouse atlas (3rd edition), to define the single functional areas. Cortical thickness of S1BF was measured from three evenly spaced MRI sections at approximate Bregma levels +0.50, −0.70, and −1.94 mm. Cortical thicknesses of AuD and DLEnt cortices were measured from sections at Bregma levels −2.06, −2.70, and −3.16 mm, and striatum thickness was measured from sections at Bregma levels +1.18, +0.50, and −0.10 mm. In S1BF, AuD and DLEnt thickness was measured from the superior border of the white matter to the pial surface of the cortex. Striatum wideness was measured from the lateral ventricle to the external capsule. For each analyzed section, we estimated six measurements (three on the left and three on the right hemisphere), resulting in a total of 18 measurements per area, which were mediated to determine the final thickness value of each analyzed area in every animal.

The article "MIM-Deficient Mice Exhibit Anatomical Changes in Dendritic Spines, Cortex Volume and Brain Ventricles, and Functional Changes in Motor Coordination and Learning" was published in 2019. Journal: Front Mol Neurosci.

### Evans Blue Injection

As terminal procedure at post-natal day P336–350, EB was injected intracerebroventricular (i.c.v.) in the mice used for the MRI follow-up study. Briefly, the animals have been anesthetized with isoflurane (5% for induction, 1.0–1.5% for maintenance, in a 70/30 N_2_O/oxygen gas mixture, 1 L/min), the head had been fixed in a stereotaxic frame, and the frontal and parietal skull bones have been revealed after a longitudinal incision of the skin: Bregma has been set as the “zero” point for all stereotaxic coordinates. Thirty minutes after anesthesia induction, 2 μL of a 0.5% solution of EB in artificial CSF were injected in the left lateral ventricle at the coordinates anteroposterior (AP) = −0.4 mm, mediolateral (ML) = 1.2 mm, and dorsoventricular (DV) = −2.2 mm, using a 50 μm glass capillary connected to a 10 μL Hamilton syringe. EB was delivered by a rate-controlled microinjector at the rate of 0.5 μL/min. After the completion of EB delivery, the injection needle remained in place for an additional 10 min for proper diffusion of the solution, and the skin was sutured back. The animals were kept under anesthesia for 2 h, then euthanized by intracardial perfusion with cold PBS followed by 4% PFA, and their brains were collected: macro photographs of the EB-injected brain have been collected.

### Statistics

All data were presented as mean ± SEM. The Shapiro-Wilk test was used to test whether datasets were normally distributed. If so, we used a Univariate Analysis of Variance test to compare two groups. The Water maze and Barnes test acquisition data were analyzed using ANOVA for repeated measures, with test day as the within-subject factor. A two-way ANOVA for repeated measurements, followed by the Sidak’s multiple comparison test, was used to analyze differences between WT and MIM KO mice at different time points in MRI analyses.

If data were not normally distributed, non-parametric tests were used to analyze the differences between experimental groups. Two Independent-samples Mann-Whitney *U* Test and Related-samples Wilcoxon Signed-Rank Test were used to compare differences between groups whose distributions did not pass Shapiro-Wilk test. Significant levels were set at *p* ≤ 0.05. All statistical analyses were performed using the IBM SPSS Statistics 24 (IBM Corp., United States). The experimenters performing behavioral testing and analyzing the histological and MRI data were blinded to the gender and genotype whenever it was possible.

The article "MIM-Deficient Mice Exhibit Anatomical Changes in Dendritic Spines, Cortex Volume and Brain Ventricles, and Functional Changes in Motor Coordination and Learning" was published in 2019. Journal: Front Mol Neurosci.

### Availability of Materials and Data

All created material and data (pictures, plasmids, analyses) are available upon request.

## Results

### MIM KO Mice Exhibit Defects in Learning and Motor Coordination

As there is a learning-associated increase in the number of new spines, we hypothesized that a regulated frequency of spine initiation is required for proper learning (Xu et al., 2009; Yang et al., 2009; Roberts et al., 2010; Fu et al., 2012). Thus, we tested whether the spine initiation factor MIM is involved in learning. MIM KO (MIM −/−) and littermate WT (MIM + / +) mice were tested at two different ages. Young mice were examined starting at age P112 ± 14 days and re-examined at P294 ± 14 days. We decided to study spatial learning with two commonly used tests: Morris Water Maze and Barnes test. We did Morris Water Maze for both age groups to be able to compare different ages. However, using the same learning test twice may affect the performance of mice at second time. Therefore, we performed Barnes test only for older cohort. We found no significant differences in MIM KO and WT mice in the water maze test when performed at a young age (Figures 1A,B,D,E). Re-testing at older age, however, showed significant impairment in spatial memory [Figure 1C, *F*(1,36) = 4.39, *p* = 0.043] and in the reverse-learning [Figure 1C, *F*(1,36) = 7.54, *p* = 0.09] in MIM KO mice when compared to WT mice. Similarly, in the probe trial, MIM KO mice performed worse than WT mice (Figures 1F,G; Probe trial *p* = 0.039, Reverse probe trial *p* = 0.047). Memory impairment was also seen in Barnes test at an age of P329 ± 14 days (Figures 1H–J, Probe trial *p* = 0.007, Reverse probe trial *p* = 0.001). In both water maze and Barnes tests, aged MIM KO mice did not discriminate between target and opposite locations in reverse probe trial (Figures 1G,J). The worse performance of MIM KO mice in spatial learning tests was not related to animal physical health. Swimming velocity did not differ between genotypes (*p* = 0.254) and there was no difference in finding a visible platform in the water maze (young – *p* = 0.535, old – *p* = 0.879) indicating that MIM KO mice saw platform normally.

To get a more comprehensive picture of how MIM affects mice behavior, we carried out a broader panel of behavioral tests (Figure 2 and Tables 1, 2). In the behaviors analyzed, we saw changes in anxiety-like behavior and social behavior, and, as shown before (Saarikangas et al., 2015), in motor coordination and strength. In the elevated zero maze test for anxiety, MIM KO mice spent significantly more time in the open arms when compared to WT mice (Figure 2A, young: *F*(1,42) = 19.60, *p* = 0.001, aged: *p* = 0.001). This behavior of MIM KO mice is indicative of a decreased level of anxiety. Accordingly, the results of the open field test showed a trend toward decreased anxiety (Figure 2B, young: *p* = 0.081, aged: *p* = 0.292) and anxiety was significantly reduced in the young MIM KO cohort in the light/dark test [young: *F*(1,42) = 14.20, *p* = 0.001, aged: *p* = 0.812]. When the depression and anxiety levels of WT and MIM KO mice were assessed in the forced swimming test, MIM KO male mice displayed a significantly reduced immobility time [aged: *F*(1,22) = 8.16, *p* = 0.009]. Furthermore, MIM KO mice exhibited impaired motor coordination when compared to WT littermates in the vertical grid test [Figures 2D,E, young: *F*(1,41) = 4.32, *p* = 0.044, aged: *p* = 0.029] and muscle weakness in the grip strength test. Muscles of MIM KO mice were weaker only in aged group [Figure 2F, young: *p* = 0.391, aged: *F*(1,39) = 11.57, *p* = 0.002]. Rota-rod test showed significantly impaired motor coordination in Young group [Figure 2G, young: *F*(1,42) = 5.23, *p* = 0.028].

The article "MIM-Deficient Mice Exhibit Anatomical Changes in Dendritic Spines, Cortex Volume and Brain Ventricles, and Functional Changes in Motor Coordination and Learning" was published in 2019. Journal: Front Mol Neurosci.

**TABLE 1:** Behavioral Characterization of young MIM KO mice.

	**Test and Parameter**	**KO vs. WT**	**WT**	**KO**	***F* Value**	***P* Value**
**Body mass**	Body mass, g	**♀↓**	21.33 ± 0.36	20.43 ± 0.37		
		**♂↓**	29.71 ± 0.72	26.60 ± 0.45		
				Genotype	*F*(1,42) = 11.68	**0.001**
				Gender	*F*(1,42) = 153.14	**0.001**
**Anxiety**	**Zero maze**					
	Distance, cm		1261.17 ± 48.86	1326.52 ± 68.70		ns
	Duration in open, s	**↑**	76.78 ± 6.49	124.33 ± 8.91	*F*(1,42) = 19.60	**0.001**
	**Open field**					
	Distance, cm		5360.59 ± 258.86	4823.80 ± 415.98		ns
	Central distance,%		32.13 ± 1.09	35.94 ± 2.58		ns
	Time in center, s		352.78 ± 23.64	464.34 ± 66.21		ns
	**Light/Dark**					
	Total distance, cm	**↓**	1847.04 ± 64.85	1594.73 ± 72.34		**0.039**
	Distance in light,%	**↑**	26.64 ± 1.17	35.15 ± 3.0	*F*(1,42) = 10.06	**0.003**
	Time in light, s	**↑**	107.83 ± 8.67	219.86 ± 34.66		**0.004**
	**Stress induced hyperthermia, °C**		1.09 ± 0.19	1.24 ± 0.22		ns
**Sensory gait**	**Nociception**					
	Hot plate, latency to reaction, s		16.37 ± 0.71	16.52 ± 0.78		ns
	**Vision**					
	Water maze visible platform		11.61 ± 2.04	10.10 ± 1.55		ns
**Motor function**	**Vertical grid**					
	Latency to top, s	**↑**	18.83 ± 2.22	30.48 ± 4.49	*F*(1,41) = 5.22	**0.028**
	**Grip strength**					
	Grip strength all paws, gf		180.15 ± 3.15	176.27 ± 5.03		ns
	**Rota Rod**					
	Time to fall, s	**↓**	186.49 ± 11.68	153.74 ± 9.24	*F*(1,42) = 5.23	**0.028**
	**Gait analysis (Foot print)**					
	Stride length, mm		73.34 ± 1.19	69.95 ± 1.57		ns
**Memory**	**Water maze**					
	Learning phase			Time	*F*(5,180) = 23.38	**0.001**
	Escape latency, s			Genotype		ns
	Probe trial					
	Target		10.99 ± 1.37	10.09 ± 1.51		ns
	Opposite	**↑**	2.68 ± 0.39	3.87 ± 0.41		**0.008**
	Left	**↑**	2.89 ± 0.37	5.64 ± 0.70		**0.001**
	Right		3.48 ± 0.45	3.78 ± 0.63		ns
	Probe trial paired test					
	Target-Opposite		*Z* = −3.92			**0.001**
				*Z* = −3.98		**0.001**
	Target-Left		*Z* = −2.63			**0.009**
				*Z* = −1.97		**0.049**
	Target-Right		*t*(25) = 5.10			**0.001**
				*t*(16) = 3.87		**0.001**
	Reverse-learning phase					
	Escape latency, s			Time	*F*(3,117) = 11.70	**0.001**
	Reverse probe trial			Genotype		ns
	Target		9.03 ± 1.05	7.63 ± 1.02		ns
	Opposite	**↑**	2.59 ± 0.50	3.87 ± 0.54		**0.023**
	Left		3.36 ± 0.46	3.63 ± 0.59		ns
	Right		4.17 ± 0.63	4.62 ± 0.88		ns
	Reverse probe trial paired test					
	Target-Opposite		*Z* = −3.87			**0.001**
				*Z* = −3.11		**0.002**
	Target-Left		*t*(25) = 5.98			**0.001**
				*t*(16) = 3.48		**0.003**
	Target-Right		*Z* = −2.70			**0.007**
				*Z* = −2.23		**0.026**
	Probe trial					
	Velocity, cm/s					ns
	Reverse probe trial					
	Velocity, cm/s					ns
**Social, psychotic**	**Pre-pulse inhibition**	**♂↓**		Genotype	*F*(1,22) = 20.68	**0.001**
	68 dB	**♂↓**	52.50 ± 4.93	28.61 ± 4.64	*F*(1,23) = 11.51	**0.003**
	72 dB	**♂↓**	58.86 ± 3.43	31.83 ± 4.98	*F*(1,23) = 21.44	**0.001**
	76 dB	**♂↓**	61.55 ± 3.36	35.11 ± 5.79	*F*(1,23) = 17.68	**0.001**
	80 dB	**♂↓**	60.99 ± 3.19	31.72 ± 6.74	*F*(1,23) = 18.50	**0.001**
	**Social dominance**					
	Total win% in tube test	**♂↓**				**0.009**
	**Forced swim test**					
	Immobility time 2–6, s	♂	165.03 ± 11.10	170.95 ± 6.95		ns

*The symbol **↑** indicates that the parameter value is significantly increased in the MIM KO mice when compared to the WT mice; the symbol **↓** indicates that the parameter value is significantly decreased in the MIM KO mice when compared to the WT mice; KO, MIM knockout; ns, statistically not significant. If the difference between genders was not significant, then data was pooled and presented as the difference between genotypes. If the difference was significant only in one gender, then it is marked in the table with a ♂ or ♀ sign next to the arrow symbol in the column “KO vs. WT.” Significant P values are highlighted with bold font.*

The article "MIM-Deficient Mice Exhibit Anatomical Changes in Dendritic Spines, Cortex Volume and Brain Ventricles, and Functional Changes in Motor Coordination and Learning" was published in 2019. Journal: Front Mol Neurosci.

**TABLE 2:** Behavioral Characterization of aged MIM KO mice.

	**Test and Parameter**	**KO vs. WT**	**WT**	**KO**	***F* Value**	***P* Value**
**Body mass**	**Body mass**, g	**♀↓**	25.17 ± 0.71	23.60 ± 0.87		
		**♂↓**	38.71 ± 1.30	30.44 ± 0.73		
				Genotype	*F*(1,36) = 17.47	**0.001**
				Gender	*F*(1,36) = 75.09	**0.001**
**Anxiety**	**Zero maze**					
	Distance, cm		834.81 ± 58.10	1048.98 ± 98.60		ns
	Duration in open, s	**↑**	52.70 ± 4.82	99.12 ± 13.14		**0.001**
	**Open field**					
	Distance, cm		3457.31 ± 266.67	3724.70 ± 221.10		ns
	Central distance,%	**↑**	30.89 ± 1.60	37.99 ± 3.04	*F*(1,39) = 5.20	**0.028**
	Time in center, s		354.54 ± 34.18	476.93 ± 71.67		ns
	**Light/Dark**					
	Distance, cm		1473.21 ± 110.25	1406.39 ± 109.44		ns
	Time in light, s		83.56 ± 10.42	96.30 ± 17.34		ns
	**Stress induced hyperthermia, °C**		1.47 ± 0.18	1.29 ± 0.12		ns
**Sensory gait**	**Nociception**					
	Hot plate, latency to reaction, s		15.00 ± 0.60	15.19 ± 1.02		ns
	**Vision**					
	Water maze visible platform		9.29 ± 1.34	9.77 ± 1.99		ns
**Motor function**	**Vertical grid**					
	Latency to top, s	**↑**	15.00 ± 1.65	26.29 ± 4.89		**0.029**
	**Grip strength**					
	Grip strength all paws, gf	**↓**	206.54 ± 2.89	185.00 ± 5.88	*F*(1,39) = 11.57	**0.002**
	**Rota Rod**					
	Time to fall, s		170.26 ± 13.22	153.71 ± 13.16		ns
	**Gait analysis (Foot print)**					
	Stride length, cm		70.53 ± 1.20	67.45 ± 1.25		ns
**Memory**	**Barnes test**					
	Learning phase Escape latency, s			Time	*F*(8,288) = 2.01	**0.045**
				Genotype		ns
	Probe trial					
	Duration in target zone, s	**↓**	15.78 ± 1.42	10.15 ± 2.84		**0.007**
	Reverse-learning phase Escape latency, s			Time		ns
				Genotype		ns
	Reverse probe trial					
	Duration in target zone, s	**↓**	12.90 ± 1.50	5.12 ± 1.60		**0.001**
	**Water maze**					
	Learning phase Escape latency, s			Time	*F*(5,180) = 10.10	**0.001**
		**↓**		Genotype	*F*(1,36) = 4.39	**0.043**
	Probe trial					
	Target	**↓**	12.90 ± 1.25	8.85 ± 1.09		**0.039**
	Opposite		3.38 ± 0.60	3.70 ± 0.75		ns
	Left		4.68 ± 0.67	4.28 ± 0.67		ns
	Right		3.90 ± 0.56	6.51 ± 1.45		ns
	Probe trial paired test					
	Target-Opposite		*Z* = −3.90			**0.001**
				*Z* = −3.11		**0.002**
	Target-Left		*Z* = −3.82			**0.001**
				*Z* = −2.10		**0.035**
	Target-Right		*Z* = −4.13			**0.001**
				*Z* = −1.35		ns
	Reverse-learning phase Escape latency, s			Time	*F*(3,180) = 24.80	**0.001**
		**↓**		Genotype	*F*(1,36) = 7.54	**0.009**
	Reverse probe trial					
	Target	**↓**	9.60 ± 1.01	6.36 ± 1.50	*F*(1,39) = 4.23	**0.047**
	Opposite		5.12 ± 0.56	6.51 ± 1.48		ns
	Left		4.69 ± 0.57	5.19 ± 0.88		ns
	Right		7.08 ± 0.84	3.82 ± 0.81		**0.021**
	Reverse probe trial paired test					
	Target-Opposite		*Z* = −2.68			**0.007**
				*Z* = −0.16		ns
	Target-Left		*t*(26) = 4.51			**0.001**
				*t*(13) = 1.40		ns
	Target-Right		*Z* = −2.01			**0.044**
				*Z* = −0.98		ns
	Probe trial					
	Velocity, cm/s		16.67 ± 0.44	15.68 ± 0.70		ns
	Distance, cm		975.33 ± 27.32	926.63 ± 42.54		ns
	Probe trial reverse					
	Velocity, cm/s		18.7 ± 0.35	17.71 ± 0.66		ns
	Distance, cm		1082.89 ± 26.34	1033.91 ± 42.61		ns
**Social, psychotic**	**Social dominance**					
	Total win% in tube test	**♂↓**	69.10 ± 6.61	30.20 ± 9.69		**0.011**
	**Forced swim test**					
	Immobility time 2–6, s	**♂↓**	180.97 ± 8.60	131.82 ± 16.91	*F*(1,22) = 8.16	**0.009**

*The symbol **↑** indicates that the parameter value is significantly increased in the MIM KO mice when compared to the WT mice; the symbol **↓** indicates that the parameter value is significantly decreased in the MIM KO mice when compared to the WT mice; KO, MIM knockout; ns, statistically not significant. If the difference between genders was not significant, then data was pooled and presented as the difference between genotypes. If the difference was significant only in one gender, then it is marked in the table with a ♂ or ♀ sign next to the arrow symbol in the column “KO vs. WT.” Significant P values are highlighted with bold font.*

The article "MIM-Deficient Mice Exhibit Anatomical Changes in Dendritic Spines, Cortex Volume and Brain Ventricles, and Functional Changes in Motor Coordination and Learning" was published in 2019. Journal: Front Mol Neurosci.

Pre-pulse inhibition of the startle response (PPI) behavioral paradigm was used to evaluate sensorimotor gating as decreased PPI is observed in schizophrenia and other neuropsychiatric disorders (Powell and Miyakawa, 2006). Young MIM KO mice had reduced PPI compared to the WT littermates (Figure 2H, see Table 1 for *p* values). We tested the mice also at the old age, however, old MIM KO mice present hearings problems, affecting the results of this test (data not shown). To test social behavior, we used the tube dominance test, which is a reliable paradigm to measure dominant behavior in male rodents to determine social ranking. The number of wins is reported as a percentage of the total number of matches. Compared to MIM KO male mice, WT male littermates at both tested ages were more dominant (Figure 2I, percentage of victories at young age: 67% WT and 33% MIM KO, *p* = 0.009; percentage of victories at old age: 70% WT and 30% MIM KO, *p* = 0.011). The results of behavioral characterization of young and aged MIM KO mice, in comparison with WT mice, are presented in Tables 1, 2.

### MIM KO Mice Exhibit a Reduced Number of Thin and Stubby Spines in the Hippocampus

We hypothesized that the hippocampal learning deficit is associated with MIM-dependent regulation of dendritic spine initiation. In order to test this hypothesis we transduced CA1 pyramidal neurons in the same mice used for behavioral analyses at P378 using a lentiviral vector carrying GFP (Figure 4A). Mice were perfused at P392, and GFP expression was visualized in brain sections stained with anti-GFP-antibodies and counterstained for DAPI (Figures 4A–C). Spine analysis of hippocampal pyramidal neurons revealed that MIM KO mice exhibit a reduced spine density of thin [WT 0.33 ± 0.03, KO 0.27 ± 0.02; *F*(1,17) = 5.54, *p* = 0.032] and stubby spines [WT 0.17 ± 0.03, MIM KO 0.08 ± 0.02; *F*(1,17) = 5.87, *p* = 0.028] in the hippocampus when compared to WT mice (Figure 4D). However, the total spine density was not affected (WT 1.70 ± 0.05, MIM KO 1.66 ± 0.08; ns).

The article "MIM-Deficient Mice Exhibit Anatomical Changes in Dendritic Spines, Cortex Volume and Brain Ventricles, and Functional Changes in Motor Coordination and Learning" was published in 2019. Journal: Front Mol Neurosci.

### MIM Is Highly Expressed in Purkinje Cells Throughout Mouse Life but in Cortex and Hippocampus Only at Early Development

We were surprised for the minor change in spine density and therefore we assessed MIM expression in different brain areas at different ages. Earlier studies have shown that MIM exhibits neuron specific expression in hippocampus (Saarikangas et al., 2015) or more generally in cerebrum (Sistig et al., 2017). In cerebellum, MIM is highly expressed in Purkinje cells and at early development (peaking at P8) in granule cells (Holst et al., 2008; Sistig et al., 2017). Strong MIM signal in internal granule cell layer started to decrease after P15 (Holst et al., 2008). Taken together, it is clear that MIM is expressed in cortex, hippocampus and cerebellum but whether expression of the MIM protein changes during development is not known. Therefore, we performed Western blotting (Figures 3A,B) and immunohistochemical (Figures 3C–N) analyses at P7, P26, P117, and P328. We first run P7 samples from WT and MIM KO mice for cortex, hippocampus and cerebellum to compare expression levels at different brain areas. All tissues had relatively high MIM expression, cerebellum expression being the highest (Figure 3A). Expression of the MIM protein in MIM KO mice was abrogated at all ages in Western blots, confirming the genotype (Figure 3A). To compare MIM expression between different ages, we run cortex, hippocampus and cerebellum samples of WT mice at same SDS-PAGE gel (Figure 3B). We run parallel samples of different animals at same age. WT mice showed a high expression of the MIM protein in the cerebellum throughout the life. The expression was lowest at P7 but relatively similar between P26 and P328. MIM expression in hippocampus was relatively high at P7 but it decreased at P26 and stayed low at later ages (Figure 3B). MIM exhibited minor expression in the cortex throughout the life. Similar to hippocampus, most expression was detected at P7 (Figure 3B). Immunohistochemistry confirmed the results from Western blot analysis. MIM showed bright staining in Purkinje cells in all ages whereas in hippocampus, MIM was detectable at P7 but not at later ages (Figures 3C–N, shown P7 and P117). Antibody staining in KO slices gave some background or unspecific staining, similar staining was obtained also when used only secondary antibodies, but Purkinje cell staining and P7 hippocampus/cortex stainings were detected only in WT mice and only when primary MIM antibodies were used. Although granule cell layer staining might be unspecific, it was reported also by other groups (Holst et al., 2008; Sistig et al., 2017) suggesting that the result shows real MIM expression at P7 in granule cells. At P7, MIM expression was restricted to mainly in somas of Purkinje cells (Figures 3D,K). Similar staining at P7 was shown also in earlier studies (Kawabata Galbraith et al., 2018). At later ages, MIM was decorating the whole dendritic tree of Purkinje cells (shown P117) (Figures 3H,M). In hippocampus at P7, MIM was expressed in pyramidal neurons in CA1-CA3 areas, granule cells in dentate gyrus and also in other MAP2 positive cells scattered throughout hippocampus.

The article "MIM-Deficient Mice Exhibit Anatomical Changes in Dendritic Spines, Cortex Volume and Brain Ventricles, and Functional Changes in Motor Coordination and Learning" was published in 2019. Journal: Front Mol Neurosci.

Because the effect of MIM deficiency in spine density was small at later age, and expression analysis do not support major function of MIM in adult mouse hippocampus, we decided to examine other possible anatomical changes in MIM KO brain. Defects in cognitive tasks, including learning, and in motor coordination, as well as decreased anxiety have been associated with schizophrenia (Powell and Miyakawa, 2006). The most typical histological changes in transgenic mice modeling schizophrenia are associated, in addition to dendritic spine density and/or morphology, with enlarged ventricle volume and decreased cortical volume (Khelfaoui et al., 2007; Ayhan et al., 2011). Thus, we next analyzed these parameters in MIM KO mice.

### MIM KO Mice Exhibit Enlarged Ventricles

Neuroimaging and postmortem studies have shown that ventricular enlargement has been observed in the schizophrenic brain, which has significant correlations with the severity of symptoms of schizophrenia (Ross et al., 2006). To examine whether MIM KO mice would show ventricle enlargement, we evaluated ventricular size in *ex vivo* brain sections and *in vivo* using magnetic resonance imaging (MRI). Histochemical analysis on brain sections was performed on the same mice used for behavioral analyses. Ventricular area measurements were performed for five slices per brain selected at different distances from Bregma (0.0, −0.5, −1.5, −2.0, −3.0), encompassing the anteroposterior extension of the ventricles (Figure 5A). The total brain area was similar in MIM KO and WT mice (Figure 5B). However, the area of ventricles in all analyzed slices was significantly larger in MIM KO mice slices than in WT mice slices [ventricle area in mm^2^: Bregma 0.0 = WT 1.3 ± 0.19, MIM KO 3.1 ± 0.20; *F*(1,15) = 36.87, *p* < 0.001, Bregma −0.5 = WT 2.4 ± 0.17, MIM KO 3.5 ± 0.31; *F*(1,17) = 9.39, *p* = 0.007, Bregma −1.5 = WT 1.5 ± 0.39, MIM KO 3.5 ± 0.42; *F*(1,12) = 11.20, *p* = 0.007, Bregma −2.0 = WT 1.2 ± 0.24, MIM KO 3.4 ± 0.72; *F*(1,10) = 9.94, p = 0.012, Bregma −3.0 = WT 0.2 ± 0.06, MIM KO 1.5 ± 0.58; *p* = 0.200, Figure 5C].

The article "MIM-Deficient Mice Exhibit Anatomical Changes in Dendritic Spines, Cortex Volume and Brain Ventricles, and Functional Changes in Motor Coordination and Learning" was published in 2019. Journal: Front Mol Neurosci.

**FIGURE 5:** MIM KO mice show ventricle enlargement. **(A)** Coronal brain slices of WT mice (on the left side) and MIM KO mice (on the right side) at different distances from Bregma (0.0, –0.5, –1.5, –2.0, and –3.0). **(B)** Total brain area was similar for MIM KO and WT mice. **(C)** The area of ventricles averaged for each slice set at different distances from Bregma was significantly bigger for MIM KO mice than for WT mice. ^∗^ denotes statistical significance: ^∗^*p* < 0.05, ^∗∗^*p* < 0.01, ^∗∗∗^*p* < 0.001. Scale bar 1000 μm.

To examine when ventricles enlarge and whether the enlargement develops during aging, we did a longitudinal *in vivo* MRI study with a separate set of fourteen mice (7 WT mice, 3 females and 4 males; and 7 littermate MIM KO mice, 4 females and 3 males) between post-natal days P84 and P168 (Figures 6A,B). Increased ventricular volume in MIM KO mice was already evident at post-natal day P84 (26.60 ± 0.39 and 12.12 ± 2.23 mm^3^ in MIM KO and WT mice, respectively), and progressed during the 2 months of the longitudinal study (Figure 6C). At day P168, the total ventricular volume of MIM KO mice was significantly increased when compared to WT littermates (29.36 ± 5.86 and 12.74 ± 1.68 mm^3^ in MIM KO and WT mice, respectively, *p* = 0.0003; Figure 6C). No statistically significant differences were observed in ventricular volume between the two hemispheres within each animal group (data not shown). Notably, within the MIM KO genotype, we observed a gender-related phenotype: 2 out of 3 MIM KO males showed a clear hyper-intense signal in the brain parenchyma (Figures 6A,B Hydro) and an increase of the total brain volume (typical of hydrocephalic brain, due to tissue swelling; data not shown), suggesting a hydrocephalic condition. These two mice were not used for the subsequent analyses. The third MIM KO male mouse analyzed – despite not presenting evident hydrocephalic features – showed a wider ventricular volume when compared to a female MIM KO. This mouse also had a hyper-intense signal in the corpus callosum, suggesting leakage of cerebrospinal fluid (CSF) from the ventricles. No such subjects were found in the MIM KO female population.

**FIGURE 6:** Longitudinal MRI analysis of ventricular volume in WT and MIM KO mice. **(A)** Representative sagittal sections throughout the brain of WT, MIM KO (KO), and MIM KO hydrocephalic (Hydro) mice. **(B)** Sagittal (top row), axial (middle row) and coronal (bottom row) reconstructed T2-weighted MRI images showing parenchyma water content and ventricular size range in WT, MIM KO, and MIM KO hydrocephalic (hydro) mice. An increment in water content and in ventricle size is evident in MIM KO transgenic mice. A distinctive severe condition is apparent in male MIM KO mice, where 2 out of 3 analyzed subjects show a clear hydrocephalic condition (Hydro). **(C)** Longitudinal measurement of ventricular volume in WT (*n* = 7) and MIM KO (*n* = 5) mice between post-natal days P84 and P168. Note that at P84 day only two MIM KO and three WT mice have been analyzed; moreover, the two hydrocephalic male mice have been excluded from the analysis of ventricle volumes at all time points. Ventricular volume was measured drawing the regions of interest (ROIs) in lateral (lv), third (3v) and fourth (4v) ventricles, and in cerebral aqueduct (aq). The ventricular volume is increased in MIM KO compared to WT mice already at day P84 and progress over time. Scatter dot plot of data with mean ± SEM are presented. ^∗^ denotes statistical significance: ^∗∗∗^*p* < 0.001. **(D)** Exemplificative macro photographs of WT, MIM KO and hydrocephalic mouse brains 2 h following Evans Blue (EB) injection in the left ventricle. Tracer distribution and putative clearance are altered in MIM KO and hydrocephalic mice, as highlighted by the accumulation of EB in the ventricles and periventricular areas in MIM KO mice. However, no tracer leakage outside the ventricles was observed in MIM KO non-hydrocephalic mice.

The article "MIM-Deficient Mice Exhibit Anatomical Changes in Dendritic Spines, Cortex Volume and Brain Ventricles, and Functional Changes in Motor Coordination and Learning" was published in 2019. Journal: Front Mol Neurosci.

At the end of the MRI study, all fourteen mice were injected with a solution of Evans Blue (EB) tracer in the left lateral ventricle and sacrificed 2 h later (Figure 6D). Macro analysis of tracer distribution showed marked differences in MIM KO mice and hydrocephalic MIM KO mice compared to WT littermates, suggesting a deficiency in fluid dynamics in the MIM KO mice. MIM KO mice presented an accumulation of EB in the ventricles and periventricular areas, whereas in WT mice the signal was visible along the spinal cord, according to the drainage flow of CSF. Hydrocephalic mice show a diffuse bilateral EB signal in the caudal brain areas, indicating that the tracer freely distributes from the ventricles into the parenchyma.

### Cilia Are Not Altered in the Ventricle or Aqueduct Walls of MIM KO Mice

We tested the hypothesis that the alteration in CSF flow is the underlying cause of the increased volume of ventricles. CSF flow impairment is often due to defects in cilia (Banizs et al., 2005), which drive the CSF flow. Furthermore, MIM has been shown to regulate ciliogenesis in mouse skin dermal cells (Bershteyn et al., 2010). Thus, we examined the density and lengths of cilia in both the lateral ventricle walls and the cerebral aqueduct. No significant differences were found in any of the studied parameters (Figure 7) between MIM KO and littermate WT mice.

The article "MIM-Deficient Mice Exhibit Anatomical Changes in Dendritic Spines, Cortex Volume and Brain Ventricles, and Functional Changes in Motor Coordination and Learning" was published in 2019. Journal: Front Mol Neurosci.

**FIGURE 7:** Cilia are not altered in the ventricle or aqueduct walls of MIM KO mice. **(A,D)** Representative coronal section of the lateral ventricle **(A)** and cerebral aqueduct **(D)**. **(B–D,F–H)** show an enlarged selected area of the lateral ventricle or cerebral aqueduct wall with acetylated tubulin staining used to measure cilia density and length. **(I)** Cilia density was calculated for each image as the number of cilia divided by the length of the ventricle edge. **(J)** To assess the length of cilia we measured the length of visible cilia with the “segmented line” tool in ImageJ. Scale bars: **(A,E)** 1000 μm, **(B,F)** 200 μm, **(C,G)** 20 μm, **(D,H)** 5 μm.

### Cortical Thickness Is Reduced in MIM KO Mice

Decrease in cortical volume has been observed in schizophrenia (Andreasen et al., 2011; Cobia et al., 2012). Thus, we assessed the effects of MIM KO on cortical thickness. Gray matter thickness analysis in cortical and subcortical areas of WT and MIM KO transgenic mice revealed a significant thinning in all analyzed regions (primary somatosensory cortex, auditory cortex, dorsolateral entorhinal cortex, and striatum) at all analyzed ages (post-natal days P112, P140, and P168) in transgenic animals (Figure 8). Significant differences were observed in primary somatosensory cortex (MIM KO: 1.09 ± 0.01; 1.06 ± 0.01; 1.07 ± 0.01 and WT: 1.22 ± 0.01; 1.18 ± 0.01; 1.19 ± 0.01 mm at P112; P140; P168, respectively, *p* < 0.0001 for genotype), auditory cortex (MIM KO: 0.81 ± 0.02; 0.80 ± 0.02; 0.77 ± 0.01 and WT: 0.95 ± 0.02; 0.92 ± 0.02; 0.91 ± 0.02 mm at P112; P140; P168, respectively, *p* < 0.0001 for genotype), dorsolateral entorhinal cortex (MIM KO: 0.74 ± 0.02; 0.73 ± 0.02; 0.72 ± 0.02 and WT: 0.84 ± 0.01; 0.85 ± 0.01; 0.85 ± 0.02 mm at P112; P140; P168, respectively, *p* < 0.0001 for genotype), and also striatum (MIM KO: 1.36 ± 0.04; 1.38 ± 0.04; 1.36 ± 0.03 and WT: 1.60 ± 0.03; 1.60 ± 0.03; 1.61 ± 0.02 mm at P112; P140; P168, respectively, *p* < 0.0001 for genotype) (Figure 8). Taken together, cortical thickness is reduced in MIM KO mice.

**FIGURE 8:** Cortical thickness measurement in WT and MIM KO mice. **(A,D)** Panels show representative T2-weighted MR images of the areas analyzed, with the approximated corresponding brain levels from the stereotaxic atlas of the mouse brain superimposed (Franklin and Paxinos, 3rd edition 2007). **(A)** Primary somatosensory cortex barrel field and striatum as measured at Bregma +0.50 mm. **(B,C)** Primary somatosensory cortex and striatum areas in MIM KO transgenic mice (*n* = 5) showed a significant reduction in thickness compared to WT mice (*n* = 7). **(D)** Dorsal area of the auditory cortex and dorsolateral entorhinal cortex as measured at Bregma –2.70 mm. An equal number of lines were manually traced on each area using a “straight line” tool in ImageJ on MRI images acquired at post-natal days P112, P140, and P168. The thickness of different areas in each brain was estimated by three measurements (at different brain levels) in triplicates (see Methods for details). Coronal levels in MRI images were matched to the corresponding plates in mouse atlas (Franklin and Paxinos, 3rd edition 2007), to define the single functional areas. **(E,F)** Auditory cortex and dorsolateral entorhinal cortex in MIM KO transgenic mice (*n* = 5) showed a significant reduction in thickness compared to WT mice (*n* = 7). Data are presented as mean + SEM. ^∗^ denotes statistical significance: ^∗^*p* < 0.05, ^∗∗^*p* < 0.01.

The article "MIM-Deficient Mice Exhibit Anatomical Changes in Dendritic Spines, Cortex Volume and Brain Ventricles, and Functional Changes in Motor Coordination and Learning" was published in 2019. Journal: Front Mol Neurosci.

## Discussion

In the present study, we performed a comprehensive behavioral and anatomical analysis of the MIM KO mouse brain, revealing previously unidentified defects. In addition, we analyzed the expression of MIM at different brain regions at different ages. Behavioral analysis of MIM KO mice revealed defects in both learning and reverse-learning (Figure 1), alterations in anxiety level and reduced dominant behavior (Figure 2), and confirmed the previously described deficiency in motor coordination and pre-pulse inhibition (Figure 2). Anatomical characterization expanded our previously reported findings, showing an association between the MIM deficiency and the decrease of Purkinje cell dendritic spine density in the cerebellum in 2-week-old mice (Saarikangas et al., 2015). Based on earlier studies we hypothesized that MIM deficiency results in decrease in spine density also in hippocampal pyramidal neurons. We further hypothesized that reduced spine density would affect spatial learning. However, we found out that MIM exhibited relatively low expression in hippocampus after early development. We further revealed that effect of MIM deficiency on hippocampal spines was very modest at old mice. Thus, it is not very plausible that decreased spine density in hippocampus is underlying the observed defects in memory. Therefore we analyzed other possible anatomical differences in MIM KO mice and revealed that MIM KO mice have enlarged ventricles and decreased cortical thickness.

Learning defects and impaired motor coordination can be connected to the enlargement of ventricles (McMullen et al., 2012). The reason underlying ventricle enlargement is still unclear: the expression of MIM in the cells lining up the ventricle walls is modest or negligible (Figure 3C and data not shown), no differences were found in the ventricle cilia density and length (Figure 7), and analysis of the ventricle walls by electron microscopy did not show any obvious changes either (data not shown). Because MIM KO mice showed altered tight junctions in the kidney (Saarikangas et al., 2011), we further hypothesized that cell-cell contacts at the level of the ventricle-brain barrier could be loose in MIM KO mice, leading to a leaking ventricle wall. This could explain our MRI data showing an increase of water content in the brain parenchyma, especially in male MIM KO mice (Figure 6). However, we could not find any obvious changes in cell-cell contacts by either confocal or electron microscopy analyses (data not shown). The altered clearance of Evans Blue in MIM KO mice may indicate a defect in the fluid dynamic of CSF in the CNS of transgenic mice. Impaired CSF clearance, due to a defect in the glymphatic system (Iliff et al., 2012) was argued to explain stagnation of gadolinium in brain ventricles after lumbar injection in idiopathic normal pressure hydrocephalus (iNPH) (Ringstad et al., 2017). This is an interesting hypothesis that could apply also to MIM KO mice, where we observed a hydrocephalic-like condition in a subpopulation of male mice, however, specific experiments should be performed to confirm the presence of defects in the glymphatic system in mice lacking the expression of MIM. MRI analyses also revealed a decrease in cortical thickness in MIM KO mice (Figure 8). Thus, the most plausible explanations for enlarged ventricles are reduced cortical volume and a deficiency in CSF fluid dynamics.

The article "MIM-Deficient Mice Exhibit Anatomical Changes in Dendritic Spines, Cortex Volume and Brain Ventricles, and Functional Changes in Motor Coordination and Learning" was published in 2019. Journal: Front Mol Neurosci.

Missing in Metastasis deficiency is clearly associated with motor-coordination and muscle weakness (Figures 2E,F, Saarikangas et al., 2015; Sistig et al., 2017; Brown et al., 2018). Motor skills and muscle weakness could originate from muscle dysfunction, instead of CNS problems. However, MIM is expressed in skeletal muscles only during the development and not at all in adult mice (Mattila et al., 2003). Furthermore, in our earlier studies, we have not found any morphological or histological defects in the muscles of MIM KO mice (unpublished). Thus, it is unlikely that the defects observed in the rota-rod and grip strength tests are of muscular origin. Deficits in the rota-rod test have been reported also in previous studies (Saarikangas et al., 2015; Sistig et al., 2017; Brown et al., 2018). In all studies, including this study, MIM KO mice were performing worse than WT mice in Rota-Rod but the magnitude varies. In Saarikangas et al. (2015), MIM KO mice became worse with aging but in this study, MIM KO mice behaved similarly at both ages. In Brown et al. (2018), MIM KO mice were performing very poor in general. In Sistig et al. (2017), WT mice improved at older age whereas MIM KO mice became worse. Behavioral testing for Saarikangas et al. (2015), was done by German Mouse Clinic, whereas the testing for this study was done in our home laboratory in Helsinki. Although the main result (MIM deficiency leads to motor-coordination defects) repeats through all studies, there are differences in the magnitude and how performance develops during aging. However, currently it is not clear where differences originate.

Schizophrenia is characterized by hallucinations, social withdrawal, and cognitive decline. Mouse models of schizophrenia show deficits in learning, social behavior and pre-pulse inhibition (Powell and Miyakawa, 2006). Similarly, in our new results, MIM KO mice showed alterations in learning abilities, the reduction in dominant behavior and pre-pulse inhibition, and increased anxiety. Schizophrenia has a strong genetic background and genetic studies have identified several genes implicated in schizophrenia, which are related to neurogenesis, neuronal migration, dendrite maturation, and synaptogenesis (Fromer et al., 2014). Decreased volumes in cortical and other brain regions have been observed in schizophrenia, as well as the decrease in the dendritic spine density (Garey et al., 1998; Glantz and Lewis, 2000). In addition, lateral ventricle enlargement is one of the most consistent brain abnormalities found in patients with schizophrenia (Del Re et al., 2016). Data of our current study show that MIM KO mice exhibit an altered spine morphology (Figure 4), thinning of cortical areas (Figure 8) and enlarged ventricles (Figure 5). Moreover, the previous studies have revealed an alteration of the dendritic tree in the Purkinje cells (Sistig et al., 2017). Similar to our new results concerning MIM KO mice, many schizophrenia single-gene KO mouse models show several histological alterations, making it difficult to estimate the exact cause underlying the observed anatomical and behavioral changes. One possibility is that a specific genetic mutation can affect many cellular processes in different cells. Alternatively, the mutation might affect a single cell process in a specific cell type and this defect leads to various secondary alterations. MIM deficit can directly affect neuronal functions (e.g., reducing synaptic density), and this can lead both to the observed behavioral deficit and to the brain edema (resulting in specific cases in a hydrocephalic-like condition). To clarify these open issues, further studies are needed, where the MIM gene is knocked-out in individual cell populations, and specific hypotheses are tested. In addition, it would be interesting, but technically very challenging, to test whether CSF diversion could ease some of the symptoms detected in hydrocephalic MIM KO mice.

The article "MIM-Deficient Mice Exhibit Anatomical Changes in Dendritic Spines, Cortex Volume and Brain Ventricles, and Functional Changes in Motor Coordination and Learning" was published in 2019. Journal: Front Mol Neurosci.

## Data Availability Statement

The raw data supporting the conclusions of this manuscript will be made available by the authors, without undue reservation, to any qualified researcher.

## Ethics Statement

The animal study was reviewed and approved by the County Administrative Board of Southern Finland.

## Author Contributions

RM was responsible for planning, performing and analyzing behavioral tests for Figures 1, 2. In addition, she did everything for Figure 4 and prepared samples for Figures 3, 5, 7. IH helped RM with behavioral testing for Figures 1, 2, and did imaging and cilia analysis for Figure 7. AV and FN planned, collected and analyzed the data for Figures 6, 8. LL carried out the ventricle and brain area analysis for Figure 5. PK performed western blot analysis of MIM expression for Figure 3. TR, AK, and VL carried out electron microscopy studies. PH conceived the theoretical ideas in this work, coordinated work, drew final conclusion and led the writing of the manuscript. All authors contributed to writing and editing of the manuscript. RM was responsible for the final layout of the figures.

## Conflict of Interest

The authors declare that the research was conducted in the absence of any commercial or financial relationships that could be construed as a potential conflict of interest.
